The article "Histone Deacetylase9 Represents the Epigenetic Promotion of M1 Macrophage Polarization and Inflammatory Response via TLR4 Regulation" was retracted in 2024. Reasons: signs of a paper mill; suspected computer-generated content; unreliable results or conclusions; concerns about the data.

# Histone Deacetylase9 Represents the Epigenetic Promotion of M1 Macrophage Polarization and Inflammatory Response via TLR4 Regulation

**DOI:** 10.1155/2022/7408136

**Published:** 2022-07-30

**Authors:** Xi Cao, Man Zhang, Hui Li, Kaiming Chen, Yong Wang, Jia Yang

**Affiliations:** ^1^Department of Circulatory, Affiliated Center of Shenyang Medical College, Shenyang, Liaoning, China; ^2^Central Laboratory of Affiliated Hospital of Shenyang Medical College, Shenyang, Liaoning, China

## Abstract

Atherosclerosis is a chronic inflammatory response mediated by various factors, where epigenetic regulation involving histone deacetylation is envisaged to modulate the expression of related proteins by regulating the binding of transcription factors to DNA, thereby influencing the development of atherosclerosis. The mechanism of atherosclerosis by histone deacetylation is partly known; hence, this project aimed at investigating the role of histone deacetylase 9 (HDAC9) in atherosclerosis. For this purpose, serum was separated from blood samples following clotting and centrifugation from atherosclerotic and healthy patients (*n* = 40 each), and then, various tests were performed. The results indicated that toll-like receptor 4 (TLR4) was not only positively correlated to the HDAC9 gene, but was also upregulated in atherosclerosis, where it was also significantly upregulated in the atherosclerosis cell model of oxidized low-density lipoprotein-induced macrophages. Conversely, the TLR4 was significantly downregulated in instances of loss of HDAC9 function, cementing the bridging relationship between HDAC9 and macrophage polarization, where the HDAC9 was found to upregulate M1 macrophage polarization which translated into the release of higher content of proinflammatory cytokines such as interleukin-1beta (IL-1*β*) and tumor necrosis factor-alpha (TNF-*α*), which tend to significantly decrease following the deletion of TLR4. Hence, this study reports novel relation between epigenetic control and atherosclerosis, which could partly be explained by histone deacetylation.

## 1. Introduction

Atherosclerosis is a chronic inflammatory response with multiple etiologies [1], which is highly prevalent in patients with rheumatoid arthritis [2]. It is triggered by the infiltration of low-density lipoprotein (LDL) into the inner membrane space and their retention under the endothelium. Oxidized low-density lipoprotein (ox-LDL) formed because of oxidation and aggregation of LDL, which exerts strong proinflammatory and immunogenic effects on the inner membrane as a chronic irritant. The ox-LDL then induces an innate immune response which results in the recruitment, migration, and differentiation of monocytes into macrophages. Macrophages show a high degree of heterogeneity by presenting different polarization states throughout the pathogenesis of atherosclerosis, namely, classic activation type M1 (proinflammatory type) and the alternative activation type M2 (anti-inflammatory type) [3]. The M1 macrophages exert proinflammatory effects through the release of cytokines such as IL-1*β* and TNF-*α*, thereby maintaining chronic inflammation leading to foam cell formation and hence promoting atherosclerosis, while the M2 macrophages perform anti-inflammatory functions by producing some relevant cytokines [4–6]. Additionally, each phenotype can be transformed into the other type [7]. Sanchez et al. [8] reported that the CD38 can be tagged as the characteristic molecule of M1 macrophages. Moreover, atherosclerosis is also linked to genetic factors where epigenetic changes had been found to play a pivotal role in its progression [9]. The nongene sequence changes because of methylation and histone modification in DNA leading to changes in the gene expression levels are termed epigenetic [10], where the histone modification can proceed via mechanisms of either acetylation or deacetylation, with the former being the most prevalent in regulating gene transcription [11]. Histone acetylation and deacetylation are primarily regulated by histone acetylases (HATs) and histone deacetylases (HDACs), respectively, which catalyze the acetylation and deacetylation reactions via lysine moiety in histone [12]. The histone in nucleosomes can be modified by acetylation to alter the binding state (tight or loose) of chromatin, which translates into either the activation or inhibition of factors and results in changes in gene expression [13]. Recent studies have reported acetylated histone as a biomarker for atherosclerosis [14]. Tikoo et al. [15] studied a comparison between New Zealand white rabbits' heart tissue, which was either fed with a high cholesterol diet, high cholesterol diet combined with atorvastatin treatment, or a control diet, where the results demonstrated that the high cholesterol group had a higher mRNA level of angiotensin-converting enzyme 2 (ACE2) in comparison to control diet group, which was envisaged to be due to effect of atorvastatin to promote histone H3 acetylation (AcH3) in the promoter region of ACE2. Furthermore, Jiang et al. [16] reported higher expression levels of histone deacetylase 7 (HDAC7) and histone deacetylase 9 (HDAC9), whereas the expression levels of P300, adenosine triphosphate binding cassette transporter A1 (ABCA1), adenosine triphosphate binding cassette transporter G1 (ABCG1), and peroxidase proliferator-activated receptor-*γ* (PPAR-*γ*) were found to decrease in atherosclerosis; moreover, HDAC9 reduction resulted in a decrease in levels of proinflammatory cytokines and significantly more M2 macrophages [17, 18]. In our previous research, the lipid-related protein NECTIN2 was discovered to serve as a potential biomarker in the progression of atherosclerosis and hence can serve as a new therapeutic entity target in its clinical prevention [19].

The article "Histone Deacetylase9 Represents the Epigenetic Promotion of M1 Macrophage Polarization and Inflammatory Response via TLR4 Regulation" was retracted in 2024. Reasons: signs of a paper mill; suspected computer-generated content; unreliable results or conclusions; concerns about the data.

The toll-like receptors (TLRs) are considered essential and play a pivotal role in the inflammatory response to coronary arterial disease (CAD) [20]. The AdaptManuscriptor molecules, namely, myeloid primary response protein (MYD88) and TIRF-related adaptor protein (TRAM), are recruited for the purpose to activate various signaling pathways including mitogen-activated protein kinase (MAPK) as well as nuclear factor-kappa beta (NF-*κ*B). The TLR4 are present on the cell membrane, where they function in recognition of different exogenous ligands which in turn results in the activation of a series of inflammatory responses via NF-*κ*B pathway. Furthermore, the inflammatory response mediated by TLR4 is upregulated by ox-LDL and hence has a pivotal role in the pathogenesis of atherosclerosis [21, 22].

During the literature search, it was discovered that both ox-LDL and LPS acted as macrophage stimuli to simulate the partial lesion model of atherosclerosis. However, previous experiments by our research group found that ox-LDL, as a stimulus of macrophages, significantly changed TLR4 expression. Therefore, further experiments were performed to investigate the impact of epigenetic changes involving acetylation and deacetylation of histones on atherosclerosis and the working mechanism of histone through TLR4 regulation to ultimately influence macrophage polarization. The experiments comprised of two parts: a human subject-based experiment and a cell line-based experiment. This study aimed to detect the expression of HDAC9 and TLR4 in different human populations followed by ox-LDL incited atherosclerosis macrophages cell line to detect whether HDAC9 could regulate macrophage polarization along with inflammatory response through TLR4 regulation, which is envisaged to provide a new idea for the treatment of the targets of atherosclerosis.

## 2. Materials and Methods

The following section provides the overall method and techniques.

### 2.1. Materials

The materials used in this study are as follows: mouse mononuclear macrophage leukemia cell line (Raw264.7, Chinese Academy of Sciences, China), Roswell Park Memorial Institute (RPMI) 1640 cell culture medium (Thermo Fisher, USA), HDAC9-shRNA and NC-shRNA (Obio Technology Corporation, Ltd. Shanghai, China), phosphate buffer saline pH 7.4 (Sigma Aldrich, USA), Triton X-100 (T8200, Soleibo, China), TLR4 inhibitor (B4935, APExBio Shanghai, China), HDAC9 (PA5–11245, 1 : 1000) and TLR4 (MAI-33380, 1 : 1000) (Invitrogen, USA, 1 : 1000), IL-1*β* (A1112, ABclonal, China, 1 : 500), CD38 (A20215, ABclonal, China, 1 : 500), TNF-*α* (A11534, ABclonal, China, 1 : 500), GAPDH (WL01114, Wanleibio, China, 1 : 10000), HRP goat anti-rabbit IgG (AS014, ABclonal, China, 1 : 10000), and fluorescent secondary antibodies A-11008 and A-21050 (Invitrogen, USA). All chemicals were used without any further processing.

The article "Histone Deacetylase9 Represents the Epigenetic Promotion of M1 Macrophage Polarization and Inflammatory Response via TLR4 Regulation" was retracted in 2024. Reasons: signs of a paper mill; suspected computer-generated content; unreliable results or conclusions; concerns about the data.

#### 2.1.1. Serum Collection and Cell Culture

A total of 80 human volunteers (40 atherosclerosis patients and 40 healthy human subjects) were recruited for this study. Blood samples were withdrawn from the elbow vein of all subjects at the Central Hospital of Shenyang Medical College between May 2019 and November 2020 (approval number: symc-20210506-02). The inclusion criteria were defined as the observation of typical angina symptoms, a definite history of old myocardial infarction, a definite history of acute myocardial infarction, and coronary angiography showing coronary artery stenosis, as stated in the diagnostic criterion for coronary heart disease in the ninth edition of *Internal Medicine*. All those patients/volunteers who were either pregnant or lactating, were suffering from infectious diseases, have underwent surgery in the recent past, have any trauma, suffering from metabolic syndrome, chronic nephritis, nephrotic syndrome, systemic lupus erythematosus, gout, rheumatic heart disease, cardiomyopathy, valvular heart disease, chronic obstructive pulmonary emphysema, asthma, and malignant diseases within the last month were excluded from the study. All recruited patients and healthy volunteers were briefed about the purpose and protocol of the study before conducting any experiments. As a next step, mouse mononuclear macrophage leukemia cells were cultured *in vitro* in RPMI 1640 medium (87%) supplemented with 10% fetal bovine serum, 1% penicillin-streptomycin double-antibody, and 2% glutamine and incubated in a cell incubator at 37°C under continuous flow of 5% CO_2_ (by volume).

#### 2.1.2. ELISA

The withdrawn blood samples were allowed to clot for two hours by keeping them at room temperature and then were centrifuged at 1000×*g* for 15 minutes at 4°C. The separated supernatant (serum) was carefully harvested using a micropipette and added to nonendotoxin. The wells were then added with 100 *μ*L aliquots of standard, blank, and samples. The plate was covered with the scaler provided in the kit and incubated for 90 min at 37°C. Following incubation, the medium was carefully decanted off followed by the addition of 100 *μ*L of biotinylated detection Ab working solution into each well, and culture plates were incubated again for one hour under the conditions briefed above. Next, the wells were carefully washed with decanted solution premixed with 350 *μ*L of sterile wash buffer for 1-2 minutes, the washing solution was decanted from each well, and the plates were dried with clean absorbent papers. The washing was carried out in triplicates. Following washing, a 1100 *μ*L of HRP conjugate working solution was then added into each well and incubated again for 30 min under previously described incubation conditions. After this incubation, each well was carefully cleared of the HRP working solution, cells were washed in pentaplicate as described before, and then 90 *μ*L of substrate reagent was added to each well, and the plates were incubated again for 15 min. Finally, 50 *μ*L of stop solution was added to each well, and the optical density (OD value) was then determined using a microplate reader (Biobase, China) at an excitation wavelength of 450 nm and emission wavelength of 520 nm. All the experimental procedures on cells were carried out in the dark.

The article "Histone Deacetylase9 Represents the Epigenetic Promotion of M1 Macrophage Polarization and Inflammatory Response via TLR4 Regulation" was retracted in 2024. Reasons: signs of a paper mill; suspected computer-generated content; unreliable results or conclusions; concerns about the data.

#### 2.1.3. HDAC9-shRNA Transfection and Experiment Grouping

The HDAC9-shRNA and NC-shRNA were transfected into macrophages during their logarithmic growth phase. Briefly, a total of 20 *μ*L of HDAC9-shRNA and NC-shRNA solutions were premixed with a cell culture medium and incubated under standard conditions of temperature and CO_2_. Following this incubation for 24 h, the cell culture medium containing transfection solution was discarded, and a fresh culture solution was added to the wells (48 h). The cell transfection was then observed under a fluorescent microscope, and the data were considered acceptable if the transfection rate was ≈70%. The groups created for the experiment included the control (Raw264.7), ox-LDL (Raw264.7 induced by 20 mg/L ox-LDL [23] for 24 h)), ox-LDL + HDAC9-shRNA (ox-LDL + HDAC9-shRNA transfection), ox-LDL+ NC-shRNA (ox-LDL + NC-shRNA transfection), and ox-LDL + TLR4 inhibitor group (ox-LDL+ TLR4 inhibitor for 24 h).

#### 2.1.4. Western Blot Analysis

The cells were collected for protein harvesting following treatments. The protein was mixed with the loading buffer at a ratio of 4 : 1, followed by heating the samples at 100°C for 5 min to induce protein denaturation. The proteins were then separated by 12% and 6% polyacrylamide gel electrophoresis under an operating voltage of 60–120 V. The proteins obtained were then transferred to the polyvinylidene fluoride membrane (PVDF) by the electrotransfer method (semidry method). The membranes were blocked by a 5% blocker solution and incubated overnight at 4°C after treatment with primary antibodies against HDAC9, TLR4, IL-1*β*, CD38, TNF-*α*, and GAPDH. The Odyssey CLx system was used for visualization using HRP goat anti-rabbit IgG.

The article "Histone Deacetylase9 Represents the Epigenetic Promotion of M1 Macrophage Polarization and Inflammatory Response via TLR4 Regulation" was retracted in 2024. Reasons: signs of a paper mill; suspected computer-generated content; unreliable results or conclusions; concerns about the data.

#### 2.1.5. Immunofluorescence Analysis

For immunofluorescence analysis, the cells were grown and cultured on coverslips, followed by discarding the culture medium. The cells were then washed thrice with sterile PBS (pH 7.4), followed by the addition of cell fixative solution to fix the cells for 30 minutes at room temperature. The cells were washed twice again with PBS, and their membranes were permeabilized with 0.1% Triton X-100 at room temperature for 15 minutes. The cells were washed with the permeabilization solution again, followed by treating the cells with a blocking solution for 30 minutes. The CD38 primary antibody (1 : 200) was then added, and cells were incubated overnight at 4°C in a humid chamber. Fluorescent secondary antibodies were then added under dark conditions for 2 h at room temperature (all subsequent operations were required to be protected from light). Next, the samples were stained with Hoechst solution for 2 min to make the nucleus visible after washing off the secondary antibody. The samples were washed again with the nucleus staining solution, PBS was added, and the cells were observed under a fluorescence microscope for CD38 expression.

#### 2.1.6. Statistical Analysis

All the experimental data obtained were statistically analyzed using SPSS (version 22.0) software. The data obtained are presented as a mean of triplicates with corresponding standard deviation (*X* ± *S*). Data were subjected to one-way ANOVA and also for estimating inter-group differences as well, while Tamhane's T2 post hoc test was performed to determine pairwise comparisons. All the graphical data/results were developed using GraphPad Prism (version 8.0) software. When required, Pearson correlation analysis for data was also performed. Statistically significant differences among/between groups were considered at *P* < 0.05.

## 3. Results

### 3.1. HDAC9 And TLR4 Expression Was Upregulated in Patients with Atherosclerosis and Atherosclerosis Cell Model of ox-LDL-Induced Macrophages

As shown in Figures 1(a) and 1(b), HDAC9 and TLR4 expressions in serum samples are significantly higher in patients with atherosclerosis compared to their expression in the serum of healthy controls (*P* < 0.05). Additionally, HDAC9 and TLR4 were positively and strongly correlated in atherosclerosis serum samples (Pearson coefficient, *r* = 0.9014) (Figure 1(c)). Similarly, in comparison to the expression in the control group, a higher expression of HDAC9 and TLR4 was found in the atherosclerosis cell models (*P* < 0.05; Figures 1(d)–1(f)).

The article "Histone Deacetylase9 Represents the Epigenetic Promotion of M1 Macrophage Polarization and Inflammatory Response via TLR4 Regulation" was retracted in 2024. Reasons: signs of a paper mill; suspected computer-generated content; unreliable results or conclusions; concerns about the data.

### 3.2. HDAC9 Promoted M1 Macrophage Polarization and the Release of Inflammatory Cytokines in the Atherosclerosis Cell Model of ox-LDL-Induced Macrophages

Western blot analysis results revealed upregulated levels of HDAC9, CD38, IL-1*β*, and TNF-*α* in the atherosclerosis cell model, compared to the levels in the control group (Figures 2(a)–2(e)). Similarly, the fluorescence intensity results of CD38 revealed that M1 macrophage polarization was significantly enhanced (*P* < 0.05, Figure 2(f), image scale of immunofluorescence: 50 *μ*m). After knocking down HDAC9, the protein expression levels of HDAC9, CD38, IL-1*β*, and TNF-*α* were significantly downregulated compared to their levels in the ox-LDL-induced group. To control the relevant factors, a lentivirus transfection (negative control) was performed on the ox-LDL-induced macrophages. The results showed that the expression levels of HDAC9, CD38, IL-1*β*, and TNF-*α* in the negative control group and the ox-LDL-induced group were similar.

### 3.3. HDAC9 Upregulated TLR4 Expression in the Atherosclerosis Cell Model of ox-LDL-Induced Macrophages

In our previous experiments, a positive correlation was found between HDAC9 and TLR4. Moreover, the experiments regarding the loss of cell function demonstrated that inhibitory HDAC9 downregulated TLR4 expression (*P* < 0.05; Figures 3(a)–3(c)).

### 3.4. HDAC9 Promoted M1 Macrophage Polarization and Inflammatory Response by Upregulating TLR4

As a result of macrophage polarization, various factors are released that either promote or suppress the inflammation [24]. The levels of HDAC9, TLR4, IL-1*β*, TNF-*α*, and CD38 were upregulated in the atherosclerosis cell model, compared to their levels in the control group. Moreover, the western blot results showed that the levels of HDAC9, TLR4, IL-1*β*, TNF-*α*, and CD38 were downregulated after HDAC9-shRNA transfection (*P* < 0.05). The levels of TLR4, IL-1*β*, TNF-*α*, and CD38 were downregulated after restraining TLR4; however, there was no significant difference in the HDAC9 protein expression (*P* > 0.05; Figures 4(a)–4(f)).

## 4. Discussion

Cardiovascular diseases rank first among all causes of disease-related deaths in the world and are considered a serious threat to human health globally. Atherosclerosis is the pathological basis for most cardiovascular diseases, and its prevention and treatment are, therefore, of great significance. In the study of atherosclerosis, while inflammation, oxidative stress, and lipid metabolism are important research areas, targeted regulation of genes has gradually become a research hotspot in recent years. The present study simulated the occurrence and development of atherosclerosis by stimulating Raw264.7 macrophages using ox-LDL to investigate the specific regulatory mechanism underlying the effect of epigenetic changes on macrophage migration and inflammatory factors.

The article "Histone Deacetylase9 Represents the Epigenetic Promotion of M1 Macrophage Polarization and Inflammatory Response via TLR4 Regulation" was retracted in 2024. Reasons: signs of a paper mill; suspected computer-generated content; unreliable results or conclusions; concerns about the data.

The pathological process of atherosclerosis mainly involves fibrosis, lipid deposition, abnormal cholesterol metabolism, and vascular wall inflammation [25]. Atherosclerosis begins with damage to endothelial cells, which translates into the activation of a series of inflammatory responses, including the release of proinflammatory cytokines, the activation of signaling pathways related to inflammation and inflammatory cell immune responses, and the release of adhesion molecules.

Activated macrophages differentiate into M1 proinflammatory and M2 anti-inflammatory macrophages, each type secreting different inflammatory factors; this heterogeneity plays a crucial role in the occurrence and development of atherosclerosis. It has been reported that the phenotype of macrophages is also regulated epigenetically [26]. Epigenetic changes regulate gene expression without changing the DNA sequence. Modification by histone acetylation is one of the methods of regulation. The acetylation of histone is in a dynamic equilibrium and under regulation by histone acetylase and histone deacetylase. Findeisen et al. [27] reported that the HDAC inhibitor trichostatin A (TSA) inhibits the proliferation of neovascular endothelial cells by inhibiting the transcriptional activity of Kruppel-like factor 4 (KLF4), suggesting that HDAC exerts a regulatory effect on atherosclerosis. Moreover, studies have indicated that rs2107595HDAC9 gene polymorphism increases the expression of HDAC9 in the internal carotid artery and regulates gene expression in the blood of patients with large vessel atherosclerotic stroke [28]. HDACs and their inhibitors might regulate the production of nitrous oxide (NO). For instance, HDAC1 could be combined with the promoter of eNOS, which impairs eNOS expression and reduces the production of NO [29]. Moreover, HDAC9 inhibits cholesterol efflux by downregulating ABCA1, ABCG1, and PPAR*γ*, which might promote the activation of macrophages, and hence, affects the occurrence and development of atherosclerosis [30]. Cao et al. [31] had shown that HDAC9 deletion could upregulate the expression of PPAR-*γ*, promote M2 macrophage polarization, downregulate the expression of M1 inflammatory genes, and inhibit atherosclerosis through chromatin remodeling. Similarly, Li et al. observed that inhibiting the transcriptional activity of KLF4, promoting the expressions of CH25H5 and LXR, and activating the KLF4-CH25H/LXR pathway could improve the reversal ability of vascular cholesterol and, thus, promote the polarization of M2 macrophages and inhibit vascular inflammation [32]. In the present study, it was observed that in ox-LDL-stimulated macrophages, the expression of HDAC9 and M1 macrophages, as well as the expression of IL-1*β* and TNF-*α* proteins, increased; however, upon knocking down the HDAC9 (transfected with HDAC9si-RNA), the expressions of M1 type macrophages and IL-1*β* and TNF-*α* proteins decreased. This suggested that HDAC9 might regulate the polarization of macrophages and the expression of IL-1*β* and TNF-*α* and, thus, might regulate the occurrence and development of atherosclerosis.

The article "Histone Deacetylase9 Represents the Epigenetic Promotion of M1 Macrophage Polarization and Inflammatory Response via TLR4 Regulation" was retracted in 2024. Reasons: signs of a paper mill; suspected computer-generated content; unreliable results or conclusions; concerns about the data.

In the inflammatory response against atherosclerosis, the activation of inflammatory pathways plays an essential role. Toll-like receptors (TLRs) are single-pass transmembrane noncatalytic proteins that represent an important class of upstream protein molecules. In the human body, TLRs are expressed mainly on the cell membrane of immune cells, such as macrophages, natural killer cells (NK cells), and lymphocytes. TLRs play a role in the immune system by directly recognizing different pathogen-related molecular patterns (PAMP) [33] in nonspecific immunity after the stressor penetrates the physical barrier of the human body. As a member of the TLR family, TLR4 is expressed mainly on the membranes of macrophages and plays an important role in the inflammatory response [34]. Besides recognizing inflammatory stressors, TLR4 also recognizes ox-LDL and further aggravates lipid stasis in macrophages. Studies [35] have reported that in mice lacking the ApoE gene, TLR4 deficiency inhibits the formation of foam cells and the expression of inflammatory factors, thereby reducing atherosclerosis. The results of the present study revealed that the expression of HDAC9 and TLR4 increased in the atherosclerotic population and ox-LDL-stimulated macrophages, both of which were found to be positively correlated. Previous studies had reported that in the mice model of skin injury, TLR4 was dynamically altered within the myeloid cells during wound healing, where the changes in the myeloid TLR4 were associated with the increased expression of histone methyltransferase and mixed lineage leukemia-1 (MLL1) [36]. Menden et al. [37] had shown that HDAC6 wild-type protein expression inhibited the acetylation of LPS-induced MyD88, as well as the acetylation in HPMEC, the co-immunoprecipitation of MyD88/TNF receptor-related factor 6 (TRAF6), and proinflammatory TLR4 signaling. In the present study, it was further revealed that the expression of TLR4 was reduced after knocking down the HDAC9 (transfected with HDAC9-shRNA) in the ox-LDL-stimulated macrophages, while the expression of TLR4 was significantly reduced after ox-LDL-stimulated macrophages were treated with TLR4 inhibitors, although the expression of HDAC9 was not statistically different from that in the group with ox-LDL-stimulated macrophages, which suggested that HDAC9 might exert a one-way regulation on TLR4.

The article "Histone Deacetylase9 Represents the Epigenetic Promotion of M1 Macrophage Polarization and Inflammatory Response via TLR4 Regulation" was retracted in 2024. Reasons: signs of a paper mill; suspected computer-generated content; unreliable results or conclusions; concerns about the data.

In summary, HDAC9 might regulate the polarization of macrophages, the release of inflammatory factors, and the expression of TLR4, although the relationship among these remains unclear. The experiments conducted in the present study further revealed that in the ox-LDL-stimulated macrophages, when TLR4 inhibitors were provided, the expression of TLR4 was significantly reduced, the polarization of M1 type macrophages reduced, and the expression of IL-1*β* and TNF-*α* proteins was decreased, suggesting that TLR4 could be used as an upstream target to regulate macrophage polarization. Additionally, it could be inferred that TLR4 might serve as an intermediate link between HDAC9 and the regulation of macrophage polarization.

## 5. Conclusion

In conclusion, epigenetic changes affect the expression of mRNA and, consequently, are involved in the occurrence and development of atherosclerosis without changing the gene sequence. The present study used ox-LDL-stimulated macrophages to simulate the atherosclerosis model and showed that atherosclerosis is related to inflammation and macrophage polarization; epigenetic modification of histone also plays an important regulatory role. Moreover, in the ox-LDL-stimulated macrophages, HDAC9 expression increased and was used as a histone regulatory target to worsen atherosclerosis, which can thus be used as an early detection biomarker for atherosclerosis. The HDAC9 is a gene for histone deacetylation-modifying enzyme, and changes in its expression cause an imbalance in histone acetylation and deacetylation, which, in turn, affects the TLR4 inflammatory pathway at the gene level. Thus, HDAC9 participates in the regulation of the occurrence and development of atherosclerosis through macrophage polarization. The present study provided useful data and experimental support for targeted therapy involving the epigenetic regulation of histone to prevent the occurrence and development of atherosclerosis. In macrophages, the histone acetylation state is not static but is rather a consequence of the continuous dynamic interaction between acetylation and deacetylation under the control of cell metabolism; however, the underlying mechanism that specifically affects this dynamic process requires further investigation.

The article "Histone Deacetylase9 Represents the Epigenetic Promotion of M1 Macrophage Polarization and Inflammatory Response via TLR4 Regulation" was retracted in 2024. Reasons: signs of a paper mill; suspected computer-generated content; unreliable results or conclusions; concerns about the data.

## Figures and Tables

**Figure 1:** HDAC9 and TLR4 protein expression levels and correlation analysis. (a) HDAC9 expression level in serum samples of control group and atherosclerosis group (ELISA), ^∗∗^*P* < 0.01. (b) TLR4 expression level in serum samples of control group and atherosclerosis group (ELISA), ^∗∗^*P* < 0.01. (c) Correlation analysis of HDAC9 and TLR4 expression in serum samples from patients with atherosclerosis (Pearson correlation coefficient, *r* = 0.9.14). (d) WB band of HDAC9 and TLR4 protein expression in RAW264.7 macrophage control group and ox-LDL group. (e) Histogram of HDAC9 protein expression in RAW264.7 macrophage control group and ox-LDL group, ^∗∗^*P* < 0.01. (f) Histogram of TLR4 protein expression in RAW264.7 macrophage control group and ox-LDL group, ^∗∗^*P* < 0.01.

**Figure 2:** RAW264.7 macrophage expression levels of HDAC9, CD38, IL-1*β*, and TNF-*α*, and immunofluorescence CD38 in the control group, ox-LDL group, ox-LDL + HDAC9-shRNA group, and ox-LDL + NC-shRNA transfection group. (a) HDAC9, CD38, IL-1*β*, and TNF-*α* protein expression WB bands in the above four groups. (b) Histogram of HDAC9 protein expression in the above four groups. (c) Histogram of CD38 protein expression in the above four groups. (d) Histogram of IL-1*β* protein expression in the above four groups. (e) Histogram of TNF-*α* protein expression in the above four groups. (f) Immunofluorescence images of CD38 protein expression in the above four groups. Blue: nucleus; red: CD38 protein; blend: blue and red overlay. ^∗∗^*P* < 0.01 (control group versus ox-LDL group), ^##^*P* < 0.01 (ox-LDL group versus ox-LDL + HDAC9-shRNA group), ^∧∧^*P* < 0.01 (ox-LDL + HDAC9-shRNA group versus ox-LDL + NC-shRNA group), ^ns^*P* > 0.05 (ox-LDL group versus ox-LDL + NC-shRNA group).

**Figure 3:** RAW264.7 macrophages: HDAC9 and TLR4 protein expression in the control group, ox-LDL group, ox-LDL + HDAC9-shRNA group, and ox-LDL + NC-shRNA group. (a) HDAC9 and TLR4 protein expressed WB bands in the above four groups. (b) Histogram of HDAC9 protein expression in the above four groups. (c) Histogram of TLR4 protein expression in the above four groups. ^∗∗^*P* < 0.01 (control group versus ox-LDL group), ^##^*P* < 0.01 (ox-LDL group versus ox-LDL + HDAC9-shRNA group), ^∧∧^*P* < 0.01 (ox-LDL + HDAC9-shRNA group versus ox-LDL + NC-shRNA group), ^ns^*P* > 0.05 (ox-LDL group versus ox-LDL + NC-shRNA group).

**Figure 4:** RAW264.7 macrophages. HDAC9, TLR4, CD38, IL-1*β*, and TNF-*α* protein expressions in the control group, ox-LDL group, ox-LDL + HDAC9-shRNA group, ox-LDL + TLR4 inhibitor group, and ox-LDL + NC-shRNA group. (a) WB band of HDAC9, TLR4, CD38, IL-1*β*, and TNF-*α* protein expression in the above five groups. (b) Histogram of HDAC9 protein expression in the above five groups. (c) Histogram of TLR4 protein expression in the above five groups. (d) Histogram of CD38 protein expression in the above five groups. (e) Histogram of IL-1*β* protein expression in the above five groups. (f) Histogram of TNF-*α* protein expression in the above five groups. ^∗∗^*P* < 0.01 (control group versus ox-LDL group), ^##^*P* < 0.01 (ox-LDL group versus ox-LDL + HDAC9-shRNA group), ^∧∧^*P* < 0.01 (ox-LDL group versus ox-LDL + TLR4 inhibitor group), ^ns^*P* > 0.05 (ox-LDL group versus ox-LDL + NC-shRNA group).

The article "Histone Deacetylase9 Represents the Epigenetic Promotion of M1 Macrophage Polarization and Inflammatory Response via TLR4 Regulation" was retracted in 2024. Reasons: signs of a paper mill; suspected computer-generated content; unreliable results or conclusions; concerns about the data.

## Data Availability

The datasets used and/or analyzed during the current study are available from the corresponding author on reasonable request.

## References

[1] Zhu Y., Xian X., Wang Z. (2018). Research progress on the relationship between atherosclerosis and inflammation. *Biomolecules*.

[2] Bhattacharya P. K., Barman B., Jamil M., Bora K. (2020). Metabolic syndrome and atherogenic indices in rheumatoid arthritis and their relationship with disease activity: a hospital-based study from northeast India. *Journal of Translational Internal Medicine*.

[3] Kavurma M. M., Rayner K. J., Karunakaran D. (2017). The walking dead: macrophage inflammation and death in atherosclerosis. *Current Opinion in Lipidology*.

[4] Wolf D., Ley K. (2019). Immunity and inflammation in atherosclerosis. *Circulation Research*.

[5] Geovanini G. R., Libby P. (2018). Atherosclerosis and inflammation: overview and updates. *Clinical Science (London, England)*.

[6] Tabas I., Bornfeldt K. E. (2016). Macrophage phenotype and function in different stages of atherosclerosis. *Circulation Research*.

[7] Sun R. Z., Fan Y., Liang X. (2018). Rapamycin and FTY720 alleviate atherosclerosis by cross talk of macrophage polarization and autophagy. *BioMed Research International*.

[8] Sanchez S., Lemmens S., Baeten P. (2018). HDAC3 inhibition promotes alternative activation of macrophages but does not affect functional recovery after spinal cord injury. *Experimental Neurobiology*.

[9] Lee D. Y., Chiu J. J. (2019). Atherosclerosis and flow: roles of epigenetic modulation in vascular endothelium. *Journal of Biomedical Science*.

[10] Mews P., Egervari G., Nativio R. (2019). Alcohol metabolism contributes to brain histone acetylation. *Nature*.

[11] Lorch Y., Maier-Davis B., Kornberg R. D. (2018). Histone acetylation inhibits RSC and stabilizes the +1 nucleosome. *Molecular Cell*.

[12] Dhar S., Gursoy-Yuzugullu O., Parasuram R., Price B. D. (2017). The tale of a tail: histone H4 acetylation and the repair of DNA breaks. *Philosophical Transactions of the Royal Society of London Series B, Biological Sciences*.

The article "Histone Deacetylase9 Represents the Epigenetic Promotion of M1 Macrophage Polarization and Inflammatory Response via TLR4 Regulation" was retracted in 2024. Reasons: signs of a paper mill; suspected computer-generated content; unreliable results or conclusions; concerns about the data.

[13] Pradeepa M. M., Grimes G. R., Kumar Y. (2016). Histone H3 globular domain acetylation identifies a new class of enhancers. *Nature Genetics*.

[14] Jiang W., Agrawal D. K., Boosani C. S. (2018). Cell-specific histone modifications in atherosclerosis (review). *Molecular Medicine Reports*.

[15] Tikoo K., Patel G., Kumar S. (2015). Tissue specific up regulation of ACE2 in rabbit model of atherosclerosis by atorvastatin: role of epigenetic histone modifications. *Biochemical Pharmacology*.

[16] Khamis A., Boutry R., Canouil M. (2020). Histone deacetylase 9 promoter hypomethylation associated with adipocyte dysfunction is a statin-related metabolic effect. *Clinical Epigenetics*.

[17] Smith J. D. (2014). New role for histone deacetylase 9 in atherosclerosis and inflammation. *Arteriosclerosis, Thrombosis, and Vascular Biology*.

[18] Oksala N. K. J., Seppälä I., Rahikainen R. (2017). Synergistic expression of histone deacetylase 9 and matrix metalloproteinase 12 in M4 macrophages in advanced carotid plaques. *European Journal of Vascular and Endovascular Surgery*.

[19] Li S., Gao Y., Ma K. (2021). Lipid-related protein NECTIN2 is an important marker in the progression of carotid atherosclerosis: an intersection of clinical and basic studies. *Journal of Translational Internal Medicine*.

[20] Roshan M. H., Tambo A., Pace N. P. (2016). The role of TLR2, TLR4, and TLR9 in the pathogenesis of atherosclerosis. *International Journal of Inflammation*.

[21] Zhang X., Xue C., Xu Q. (2019). Caprylic acid suppresses inflammation via TLR4/NF-*κ*B signaling and improves atherosclerosis in ApoE-deficient mice. *Nutrition & Metabolism (London)*.

[22] Luque-Martin R., Van den Bossche J., Furze R. C. (2019). Targeting histone deacetylases in myeloid cells inhibits their maturation and inflammatory function with limited effects on atherosclerosis. *Frontiers in Pharmacology*.

[23] Pirillo A., Norata G. D., Catapano A. L. (2013). LOX-1, OxLDL, and atherosclerosis. *Mediators of Inflammation*.

[24] Wang Z., Wu L., Pan B., Chen Y., Zhang T., Tang N. (2021). Interleukin 33 mediates hepatocyte autophagy and innate immune response in the early phase of acetaminophen-induced acute liver injury. *Toxicology*.

[25] Xu S., Kamato D., Little P. J., Nakagawa S., Pelisek J., Jin Z. G. (2019). Targeting epigenetics and non-coding RNAs in atherosclerosis: from mechanisms to therapeutics. *Pharmacology & Therapeutics*.

[26] Stillman B. (2018). Histone modifications: insights into their influence on gene expression. *Cell*.

[27] Findeisen H. M., Gizard F., Zhao Y. (2011). Epigenetic regulation of vascular smooth muscle cell proliferation and neointima formation by histone deacetylase inhibition. *Arteriosclerosis, Thrombosis, and Vascular Biology*.

The article "Histone Deacetylase9 Represents the Epigenetic Promotion of M1 Macrophage Polarization and Inflammatory Response via TLR4 Regulation" was retracted in 2024. Reasons: signs of a paper mill; suspected computer-generated content; unreliable results or conclusions; concerns about the data.

[28] Manea S. A., Vlad M. L., Fenyo I. M. (2020). Pharmacological inhibition of histone deacetylase reduces NADPH oxidase expression, oxidative stress and the progression of atherosclerotic lesions in hypercholesterolemic apolipoprotein E-deficient mice; potential implications for human atherosclerosis. *Redox Biology*.

[29] Leucker T. M., Nomura Y., Kim J. H. (2017). Cystathionine *γ*-lyase protects vascular endothelium: a role for inhibition of histone deacetylase 6. *American Journal of Physiology. Heart and Circulatory Physiology*.

[30] Zhang J., Xu Z., Gu J. (2018). HDAC3 inhibition in diabetic mice may activate Nrf2 preventing diabetes-induced liver damage and FGF21 synthesis and secretion leading to aortic protection. *American Journal of Physiology. Endocrinology and Metabolism*.

[31] Cao Q., Rong S., Repa J. J., St Clair R., Parks J. S., Mishra N. (2014). Histone deacetylase 9 represses cholesterol efflux and alternatively activated macrophages in atherosclerosis development. *Arteriosclerosis, Thrombosis, and Vascular Biology*.

[32] Li Z., Martin M., Zhang J. (2017). Krüppel-like factor 4 regulation of cholesterol-25-hydroxylase and liver X receptor mitigates atherosclerosis susceptibility. *Circulation*.

[33] Wang K. L., Chen S. N., Huo H. J., Nie P. (2021). Identification and expression analysis of sixteen Toll-like receptor genes, TLR1, TLR2a, TLR2b, TLR3, TLR5M, TLR5S, TLR7-9, TLR13a-c, TLR14, TLR21-23 in mandarin fish Siniperca chuatsi. *Developmental and Comparative Immunology*.

[34] Kang D. Y., Sp N., Jo E. S. (2021). Non-toxic sulfur inhibits LPS-induced inflammation by regulating TLR-4 and JAK2/STAT3 through IL-6 signaling. *Molecular Medicine Reports*.

[35] Kalchiem-Dekel O., Yao X., Barochia A. V. (2020). Apolipoprotein E signals via TLR4 to induce CXCL5 secretion by asthmatic airway epithelial cells. *American Journal of Respiratory Cell and Molecular Biology*.

[36] Frank M. (2019). Histone methylation directs myeloid TLR4 expression and regulates wound healing following cutaneous tissue injury. *Journal of Immunology*.

[37] Menden H., Xia S., Mabry S. M. (2019). Histone deacetylase 6 regulates endothelial MyD88-dependent canonical TLR signaling, lung inflammation, and alveolar remodeling in the developing lung. *American Journal of Physiology. Lung Cellular and Molecular Physiology*.

